This article has been retracted.

# Closed Home Physical Education Teaching Model and Response Strategies Based on Big Data Technology

**DOI:** 10.1155/2022/7670725

**Published:** 2022-08-31

**Authors:** Guohong Xu

**Affiliations:** Institute of Physical Education, Ludong University, Yantai 264025, China

## Abstract

Online teaching is carried out nationwide in the context of the new crown epidemic prevention and control, and physical education, as one of the compulsory courses in schools and universities, is included within the content of online line lessons. Online physical education teaching is a new approach and attempt to switch from an auxiliary teaching tool to the main teaching tool. The subject matter, target audience, teaching methods, and content of physical education classes have changed dramatically. The development of online physical education has played an important role in popularizing the concept of “sports for life” and establishing the concept of lifelong exercise. Through the analysis and research on the characteristics of online physical education, we propose the measures to promote the overall online teaching ability and level of physical education teachers in the postepidemic period, gradually promote the reform of online and offline physical education, and promote the integration of school physical education and social sports, as well as to build a physical education teacher training system that integrates online and offline development and improve and strengthen the management of Internet physical education resources. Since the teaching effect of online teaching is limited by the teaching means and content, which leads to the low accuracy of the evaluation of online sports teaching effect, for this reason, this paper designs a model based on big data technology and artificial intelligence algorithm for enhancing closed home sports teaching, obtains the overall situation of online physical education by using convolutional neural network to process physical education video sequences, and improves the system performance by embedding the algorithm into the big data framework, to avoid the interference of teaching environment and complete the evaluation of high precision online sports teaching effect. The experimental results show that the proposed method evaluation can improve the computing rate based on ensuring the high accuracy evaluation of physical education online teaching effect.

## 1. Introduction

In 2020, in the face of the sudden new crown pneumonia epidemic, China's Ministry of Education reacted quickly according to the real-time situation and issued a notice about the postponed start of the spring semester of 2020, deciding to postpone the start of schools of all levels and types, encouraging localities to use the Internet and information-based educational resources to provide learning support for students, ensuring that classes are suspended without stopping, doing everything possible to reduce the negative impact of the epidemic on students and giving out guidelines for online teaching. A nationwide online teaching campaign was quickly launched [1–3].

Although physical education as a basic, compulsory subject has its own subject-specific, conditional, and geographical requirements, it is also important to overcome external objective factors to ensure the smooth conduct of physical education classes within the limits of our ability, so that students can perform physical exercises and meet physical fitness standards as much as possible within their home environment. The outline of building a strong sports nation states that fitness activities for all should be widely carried out and that they should be carried out according to time and place and according to need. Therefore, online physical education is in line with the general policy of the country and is conducive to the gradual penetration of physical exercise and health awareness into people's daily life and work, and the realization of sports for life. The significance of home-based online physical education is shown in Figure 1.

With the development of the epidemic prevention and control war, the Party and the State are highly concerned about people's life and health safety, and a series of epidemic prevention measures are being carried out, among which “home quarantine” is one of the important measures, which requires residents to purchase daily necessities and seek medical care, and other residents are required to stay at home and not go out, except for basic activities such as purchasing necessities and seeking medical care [4–7]. During home isolation, the Ministry of Education requires schools of all levels and types to carry out teaching tasks and home study guidance online. China has 518,800 schools of all levels and types, 16,728,500 full-time teachers, and 276 million students. The education system's large-scale online education for the nation's hundreds of millions of students during the epidemic's prevention and control is an unprecedented initiative in history and the first of its kind in the world.

The nationwide online physical education is also a precedent in the history of physical education in China, which shows that online physical education, as a new teaching method, is an inevitable product of today's network information era and is a necessary path for China's teaching to become technological and modernized. Online physical education is converted from teachers and students sharing the same space to teachers and students belonging to different spaces under the conditions of epidemic prevention and control, from 3D three-dimensional teaching by word and body to 2D flat teaching and physical education action skills video display through online teaching platforms (Tencent Conference APP, Tencent Classroom APP, Nail APP, and so on), from face-to-face teaching in the same place and space at the same time to live classes or prescribed time periods for learning [8–12].

The video class is converted from teaching aids to main teaching means. The above five conversions are the passive development of online physical education in response to the new epidemic, which has accumulated valuable experience for the development of online physical education in China, while responding to the Ministry of Education's policy of “suspending classes without stopping school” and minimizing the impact of the epidemic on students. Online teaching is the result of the accumulation of basic resources of education informatization, which accelerates and reconstructs an all-media physical education learning ecology.

The connotation and performance of lifelike sports are the penetration of sports and fitness activities into daily life and their close integration with daily life, becoming the fifth element of life in addition to clothing, food, housing, and transportation, becoming a new way of life and an important feature and an important way to achieve high quality of life. The lifestyle of sports is a social phenomenon that emerges along with the process of modern civilization, and people establish a healthy and active lifestyle, which is a concrete manifestation of people taking sports activities as an organic part of their lives and making them an important part of their lives. Sports lifestyle means the integration of sports factors into the way of life and production, where sports factors do not refer to simple sports skills but to sports habits, sports ways, etc. For example, daily trips are mainly cycling and walking, family members regularly organize sports or watch sports competitions together, sports expenses and sports closely related expenses as fixed expenses in the daily production expenses of the family, essential physical fitness exercise. The diversification of sports information dissemination is an important manifestation of the living of sports. Along with the rapid development of science and technology and the arrival of the era of self-media for all, sports information, as a kind of information resource, quietly penetrates people's daily life and influences their lifestyles and attitudes [13]. The dissemination of sports-related information ranges from the initial mainstream media such as TV, newspapers, and radio to sports-related applications nowadays. Sports groups range from professional athletes to mass amateurs and from children to the middle-aged and elderly.

Many examples prove that the diversification of sports information dissemination is also one of the important features to promote the popularization of sports life. Nowadays, the living standard of Chinese residents has been improved substantially, the people's demand for material and cultural life is increasing, the number of people participating in physical exercise has increased significantly in recent years, and the people's demand for a healthy life and a high quality of life is getting higher and higher. From participation in sports activities in previous years under the call of unit organizations, to the emergence of a large number of social sports group organizations such as running teams, teams, mountain climbing teams, and the rise of related events, from passive participation to active seeking exercise, people's mass participation in sports is increasingly active, and the frequency of participation has gradually developed from random irregularity to stability, periodization, and normalization.

The era of big data has opened a major transformation and social change. As an information technology and service industry that discovers new knowledge, creates new values, and enhances new capabilities, big data technology not only gives new meaning and value to many basic data, but also gradually becomes the main driving force for deep-level adjustment and optimization of social structure, social functions, and social actions. Under the influence of this background, the school education field, which is closely related to big data, has also accelerated the pace of turning to the smart education model. In the era of smart education, physical education still faces many bottleneck problems, which seriously limit the effective release of the value benefits of physical education series [14]. It is particularly worth studying whether we can use the advantages of big data technology to crack some difficult problems faced by physical education, improve and optimize the quality and effect of physical education, and further deepen the pace of physical education reform in Chinese schools.

The evaluation of the teaching results in traditional physical education classrooms is mainly through the comprehensive evaluation of students' usual homework completion and regular examinations and assessments, which has one-way and closed characteristics. Through scientific analysis of accurate and effective big data, we can not only observe single students' mastery of the knowledge system of this course vertically, but also compare the learning situation of students of the same major horizontally and compare and judge students' ability in listening, reading, writing, and translating in all aspects. It breaks the limitation of the traditional teaching evaluation system, which mainly relies on exam scoring, and through data analysis and collection, it can customize personalized learning reports for each student, inspire students to establish goals and make learning career plans, which truly reflects the directivity and guidance of teaching evaluation. The influence of big data in the teaching process: the sports classroom in the postepidemic era integrates big data analysis into the three links before, during, and after class, breaking the closed-loop operation of traditional teaching and shaping a new open and interactive teaching platform, allowing teachers and students to communicate unhindered and showing infinite vitality [15, 16, 17].

The main contributions of this paper are as follows. Firstly, we analyze that although online physical education in higher education institutions is extremely important for maintaining students' physical and mental health during the new crown pneumonia epidemic, the narrow home space, difficulty in effectively monitoring course learning and insufficient preparation for online teaching, low IT literacy of physical education teachers, and unclear objectives of online physical education have made online physical education fail to achieve the expected teaching effectiveness. To this end, this paper proposes a closed home-based physical education teaching model based on big data and artificial intelligence algorithms for improving online physical education model, improving physical education teachers' IT literacy, and clarifying physical education goals, which provides a reference for better promoting the development of online physical education and the construction of a new physical education model.

## 2. Related Work

### 2.1. Enclosed Home Physical Education

Traditional physical education is mainly outdoor, students are engaged in physical activities under the guidance of teachers, and the natural teaching environment affects the quality of physical education and teaching effect impact. The most important feature of physical education teaching is that the teacher in the classroom is organized to guide the students' learning and practice, and the teacher's face-to-face explanation of techniques, movement demonstration, and error correction are the main features. During the epidemic, the teaching site was transferred from outdoor to home, and the learning environment of students changed. Teachers became online video instructors across the air, and students became online observers and offline independent practitioners [18, 19]. The change in the teaching venue, the passive acceptance of home online physical education by individuals, the psychological environment of student learning needs to adapt, and teachers and students cannot intuitively grasp the learning effect like traditional physical education. Then again, the limited space at home, the traditional sports venue equipment, and sports equipment cannot be used properly, which makes many physical sports teaching activities with high demand for venue cannot be carried out normally, such as group co-court confrontation projects basketball and soccer, which also affects the actual teaching effect.

The teaching method of physical education under the new crown pneumonia epidemic changes the traditional physical education teaching mainly in the way of teachers transmitting verbal information to teach students theoretical knowledge of sports and instruction of sports technology in verbal language, which can effectively grasp the stage of skill learning, and timely error correction and explanation and demonstration [20–22]. This way of transmitting verbal information is also an important way of communication between teachers and students. The traditional way of teaching physical education has the use of organizing mutual communication and collaboration between students in the practice process to develop their collectivism. In sports where competition is the main activity, teamwork can be developed. Online physical education is clearly different from traditional physical education.

Online physical education is based on students' independent learning style, which places higher demands on teachers to organize teaching online, anticipate students' learning progress, correct errors online, and teach at different levels. The transition from skills-based teaching and basic fitness-based content to traditional martial arts and basic fitness-based online teaching at home requires students to exercise at home consciously, which is conducive to personalized teaching and the development of students' independent thinking skills. Outdoor face-to-face becomes online teaching across the screen, which cannot control the effect of students' independent learning. The adoption of online teaching combined with offline teaching will increase teachers' personal workload, and the preparation of lessons should be more adequate. Compared with the traditional offline teaching method, online teaching requires more preparation for lessons, online live teaching and recorded teaching videos, online Q&A, and online homework correction after lessons, which invariably increases teachers' teaching difficulty [23].

Table 1 shows that 88.37% of teachers took online live and recorded teaching. As one of the teaching contents in secondary schools, physical education is also an examination content, and in the context of the epidemic, it is especially important to develop physical exercise and enhance physical fitness. Under the requirement of the Ministry of Education to suspend classes without stopping school, physical education is carried out in an orderly manner, and most of them take online live or recorded online teaching forms. The development of online physical education at home is shown in Table 1.

The large-scale online home physical education practice is not only an emergency measure in the face of the epidemic, but also a test of “Internet+” physical education, and an effective means to promote the information of education and teaching and help students develop lifelong physical education learning. To understand the situation of online physical education at home for junior high school students, this paper investigates the current situation of online physical education at home for students and uses a questionnaire to study the basic situation of online physical education, the impact of online physical education at home on teachers' teaching and students' learning, and teachers' and students' self-evaluation of physical education at home and learning [24–27]. While online physical education during the epidemic effectively expanded the content, time, and space of university public physical education courses, online physical education courses can effectively update and deliver the physical education knowledge needed by university students in response to the problems of insufficient hours of university physical education theory courses and teachers' shortage in theory teaching. During this epidemic, some universities have incorporated a part of the knowledge of immunity boosting against the epidemic, sports, and health into the online sports courses and enriched the teaching content by providing students with health education related sports theory knowledge and project related physical fitness exercises as a necessary supplement to the online courses. This also makes the teaching of physical education theory classes clearer, more graphic, and vivid and also greatly stimulates students' interest in online learning.

### 2.2. Big Data Technology

In the era of rapid development of big data, big data technology is widely used in all aspects of society, and the data information in the Internet is now exploding [28]. At present, with the intelligent development of big data technology, the data of home online physical education continues to grow exponentially with positive correlation, and the frequency of using home online physical education sharing platform also continues to grow. Faced with the situation of massive data of home online physical education, how to manage these massive data efficiently and explore the value of home online physical education has become the current problem faced by the home online physical education sharing platform [29, 30]. To make the home online physical education sharing platform meet the needs of users and provide them with accurate services, it is obvious that traditional technology can no longer meet its application. In the current big data environment, the technical processing based on Hadoop cloud platform can maximize the mining of massive data and provide clear data information for the home online sports teaching sharing platform using MapReduce parallelization model, thus meeting the current demand of archival users for both simplified retrieval procedures and precise access to online sports teaching that needs to be found.

Hadoop cloud platform core technology of MapReduce: Hadoop is a distributed system open-source framework developed by the Apache Foundation. Hadoop is a theoretical framework with good high performance, high reliability, and fault tolerance realized based on Google cloud computing. Hadoop system is a system specifically for large-scale data processing; the system can effectively understand users' feedback information about information resources, meet users' requirements of finding and using information resources in a distributed space, and form a good interactive model. Hadoop, as a storage and computing platform for large-scale data, can not only integrate heterogeneous data distributed in different domains on a single platform, but also store data effectively, improve retrieval efficiency, and avoid useless retrieval and MapReduce is one of the core technologies of the Hadoop cloud platform, and Hadoop is based on Google's development of an open-source MapReduce computing framework for handling parallel computing of big data. In the operation of MapReduce, its simplification parallel computing can be very useful for high-performance application requirements, reducing the difficulty of use when the user retrieves and speeding up the data analysis and processing capabilities, so it is widely used in the field of data mining [31, 32]. MapReduce divides data processing into two parts: the first part is the mapping Map, and the second part is the simplification Reduce. In simple terms, MapReduce big data technology first decomposes the user input data into *M* small data sets in the Map mapping part, and these *M* small data sets correspond to *M* Map tasks, which are processed separately for the decomposed data, and the results are finally obtained by aggregating the results in the second part of Reduce. In the large-scale home online physical education data, the use of MapReduce big data technology of Hadoop cloud platform can not only improve the performance and reliability of the sharing platform, but also meet the user's grasp of the accuracy of the acquired data, and most importantly, Hadoop makes up for the deficiency of the home online physical education sharing platform in the integration of data and information resources.

The establishment of the home online sports teaching sharing platform needs to meet the characteristics of its own platform and meet the use of different browsers such as PC, cell phone, and mobile end, so the optimization of data processing and data mining technology of the home online sports teaching sharing platform is crucial. According to the continuous optimization of big data technology, the home-based online physical education sharing platform realizes efficient interoperability of home-based online physical education with the help of the current optimized technology and personalizes the service method of the home-based online physical education sharing platform. Therefore, the home online physical education sharing platform must meet its own development needs based on big data technology.

The structure deployment of the home online physical education sharing platform: the goal of the home online physical education sharing platform is to facilitate the use of archival resources, diversify online physical education services, efficiently manage online physical education resources, and optimize archival data processing and mining technology. The construction of the platform will be efficient, interconnected, interoperable, and shared. At the beginning of the construction of the home online physical education sharing platform, due to the incomplete application of technology, limited users, and low level of resource management, the users are only limited to internal users, for which the comprehensive performance of the platform is not high enough, and its application server, database processing and mining server, and resource management server all run on one server. However, with the development and continuous maturity of big data technology, the range of users is expanding, causing the length of access to the server to lengthen and slow down. As the shared platform stores more and more data resources, this requires the application server, database server, and information resource management server to be deployed independently. The application scope of the platform cannot be limited to PC users, but to meet different user needs to enhance the diversity of online physical education services, which requires the performance of the platform to be improved accordingly and requires the introduction of advanced big data technology and the use of Distributed system to solve the problem of the increase of big data resources and the performance of high concurrent data, from the traditional single structure deployment to the efficient structure deployment of multiple distribution.

## 3. Methods

### 3.1. Model Architecture

The overall framework of the closed home physical education model is shown in Figure 2. The framework mainly consists of two steps: part 1, segmentation recognition of continuous action sequences by using a fixed length sliding window, to circumvent the disadvantage of poor recognition of transition actions by sliding windows, only nontransition actions are trained for recognition here, and finally, the dynamic actions and physical education actions in complex continuous actions are calibrated. In the second part, the boundaries of physical education actions (sitting, standing, and lying) are detected, the transitional actions existing between the two types of physical education actions are calibrated, and then, the class of transitional actions existing between action states can be determined according to the finite state machine.

### 3.2. Big Data Technology

The establishment of a home online physical education platform requires a database adapted to the big data environment. At present, Hadoop is the most common data storage technology, which is suitable for large-scale data storage and management. The improvement of data storage and management technology is paving the way for data retrieval. In the retrieval function of the home online physical education platform, the data storage and statistical analysis of home online physical education are the foundation of the platform. The analysis and calculation stage in the data retrieval function can be realized by using MapReduce, which is to divide the data to be processed into individual small data and process them separately in parallel, with the following operation process: there are two types of nodes in MapReduce, namely, the management task *JobTracker* and the execution task *TaskTracker*. *JobTracker* is the manager and is responsible for scheduling and monitoring the execution of *TaskTracker*, which assigns tasks and gives Map and Reduce functions to idle *TaskTracker* for execution. The parallel algorithm of MapReduce is to achieve the clustering of Map and Reduce, the system will plan the input data into a certain size of file blocks, Mapper will process each file to achieve the first stage of clustering, and then, a single Reduce processes the data from the first stage of clustering to achieve the second stage of clustering, an algorithm executed with several Mappers and a single Reduce.

### 3.3. Key Frame Extraction

The behavioral states described by key physical education actions in video sequences are more meaningful for analyzing and recognizing human behavior and for reducing data redundancy and computational load. This paper proposes a key frame extraction method based on an improved Gaussian mixture model. In the traditional Gaussian mixture model, the learning rate is fixed during the learning process, so the weights of the Gaussian distribution corresponding to the motion target will rise after a certain time and gradually update to the background distribution, which will lead to the appearance of holes and then disappearance of the motion target, especially the target with slow motion speed. Therefore, in this paper, the velocity *v* of the moving target is associated with the learning rate *a*_*x*,*y*,*t*_ of the pixel points, which is dynamically adjusted as a dynamic variable. The motion velocity *v*_*x*,*y*,*t*_, defined in this paper, of the mathematical expression is shown in equation. Using this method for motion target detection effectively improves the operation speed and enhances the dynamic environment ground adaptivity. The coarse segmentation flow chart is shown in Figure 3.

(1) $$\begin{array}{c} \left\{\begin{array}{c} u_{x,y,t}=O_{x,y,t}D/\Delta t\\ \sqrt{{\left(y_{t}-y_{t-1}\right)}^{2}+{\left(x_{t}-x_{t-1}\right)}^{2}} \end{array}\right., \end{array}$$

where Δ*t* represents the time interval and is a fixed value. *x*_*t*_ and *y*_*t*_ refer to the rank order of the center pixel points of the smallest outer rectangle of the set of moving target points in frame *t*. For the set of foreground pixel points composing the moving target, the velocity *v*_*x*,*y*,*t*_. y of each of these points is represented by the same velocity value. To prevent a fixed update rate from recognizing low-speed targets as background, the learning rate *α*_*x*,*y*,*t*_ needs to be dynamically adjusted with the change in velocity *v*_*x*,*y*,*t*_. For a high-speed target, it does not stay in a fixed region, and there is no gradual conversion of the foreground distribution to the background distribution, so the pixel points need to maintain a stable, high learning rate; the exact opposite is true for a low-speed target. The formula that defines the learning rate *α*_*x*,*y*,*t*_ is shown as follows:

(2) $$\begin{array}{c} \alpha_{x,y,t}=\left\{\begin{array}{c} \frac{U_{x,y,t}}{u_{x,y,t}+\gamma^{\text{'}}},\\ \alpha_{x,y,t-1}. \end{array}\right. \end{array}$$

In the equation, *v*_0_ denotes the velocity critical threshold, which is used to distinguish the motion target with high speed from low speed. A pixel point's learning rate is initialized to the initial value *α*_*x*,*y*,*t*_ when it satisfies the following conditions: (1) the distribution model matched at moments *t-*1 and *t* has changed; (2) the velocity is zero for 5 to 10 consecutive frames.

### 3.4. Null Convolutional Neural Network

MIMU measurements have noise, and different operating temperatures bring bias error, the MIMU measurements are modeled as u_*n*_^*IMU*^ subscript *n* is the time window, and the angular rate *ω* and acceleration measured at high frequencies are modeled to introduce noise and bias error:

(3) $$\begin{array}{c} u_{n}^{\text{IMU}}=\left(\begin{array}{c} \omega_{n}^{\text{IMU}}\\ a_{n}^{\text{IMU}} \end{array}\right)=G\left(\begin{array}{c} \omega_{n}\\ a_{n} \end{array}\right)+b_{n}+w_{n}, \end{array}$$

where *b*_*n*_ is the constant bias error, *w*_*n*_ is the Gaussian white noise with zero mean, and *ω* is the gyroscope measurement:

(4) $$\begin{array}{c} a_{n}^{\text{IMU}}=C_{n}^{b\text{T}}\left(\frac{\left(v_{n}-v_{n-1}\right)}{\text{d}t-g}\right), \end{array}$$

where *a*_*n*_^IMU^ is the linear acceleration excluding gravity in the navigation coordinate system, *v*_*n*_ is the MIMU measured velocity value in the navigation coordinate system, and *G* is the intrinsic calibration matrix:

(5) $$\begin{array}{c} G=\left(\begin{array}{cc} S_{\omega }M_{\omega } & A\\ 0_{3\times 3} & S_{a}M_{a} \end{array}\right)\approx I_{6}. \end{array}$$

DCNN injects voids in the convolutional layer compared with the standard CNN, which can perceive more information and reduce the number of operations while keeping the parameters of the convolutional layer unchanged. A DCNN is studied and constructed to compensate the angular velocity of the gyroscope output to eliminate errors and drift. The input of the DCNN is the data collected from the MIMU in the window N; i.e., ∑_*N*=0_*u*_*n*−*N*_^*IMU*^, *N*, *N* is defined as the convolution kernel size multiplied by the maximum value of the expansion gap, the sampling rate is 100 *Hz*, and the output is the gyroscope correction *ω*_*n*_. The model is cascaded with five convolution blocks, and the parameters of each convolution layer are set in Table 2.

The DCNN flow chart is shown in Figure 4. A batch normalization (BN) operation layer and a smooth Gaussian error linear unit (GELU) activation function are inserted before and after the two convolutional layers of the CNN. The main role of the BN layer is to eliminate the error accumulation of singular samples, and the input data distribution in each layer of the CNN will be affected with the training parameter update of the previous layer. The BN layer GELU is a high-performance neural network activation function whose nonlinear variation is a kind of expected stochastic regular transformation, and the random errors inherent in MIMU MEMS accelerometers and gyroscopes are approximately Gaussian distributed. U activation function can enhance the model learning capability more effectively.

### 3.5. Fusion Data

The fused gyroscope P.E. action angle estimate: $\alpha_{g}=\left[\begin{array}{c} \theta_{g}\gamma_{g}\psi_{g} \end{array}\right]$, and accelerometer and magnetometer P.E. action angle estimates: $\beta_{g}=\left[\begin{array}{c} \theta_{a}\gamma_{a}\psi_{a} \end{array}\right]$, with the initial yaw angle determined by the magnetometer. Using the estimated gyroscope P.E. action angle after DCNN correction as the predicted state value and the angle obtained from the accelerometer and magnetometer as the measured value, the established EKF state equation and measurement equation are as follows:

(6) $$\begin{array}{c} \left\{\begin{array}{c} x_{k}=\Phi x_{k-1}+\Gamma W_{k-1},\\ Z_{k}=Hx_{k}+V_{k}, \end{array}\right. \end{array}$$

where *k* is the moment value, **x**_*k*_ is the state value, **Z**_*k*_ is the measurement value, Φ is the state transfer matrix, Γ is the noise driven matrix, *H* is the measurement transfer matrix, *W*_*k-1*_ is the system noise driven matrix, and *V*_*k*_ is the measurement noise matrix, satisfying the mean value of zero and the variance array of uncorrelated white noise *Q* and *R*, respectively.

## 4. Experiments and Results

### 4.1. Experiment Setup

In this paper, the behavior recognition dataset NTU-RGB + *D* established by a physical education laboratory in China is used as the experimental data. The dataset consists of 60 physical education action categories (divided into three categories of daily physical education actions and two-player interaction behaviors) and 56,880 video physical education action samples, and each video contains one physical education action, including single physical education actions (e.g., sitting) and two-player physical education actions (e.g., shaking hands with each other). There are also four different forms of PE teaching action data: RGB video, 3D skeleton data, depth map sequence, and infrared video. In this paper, 3D skeleton data is chosen for the study of behavior recognition based on skeletal information.

The experimental environment is Windows l0 operating system; CPU is Intel(R) Core (TM) i7-9750H; GPU is GeForceGTX1650. Design network is implemented using PyTorch deep learning framework. The big data nodes are configured as follows: in the experiments, the data cluster used is composed of 27 nodes, including one main node, one scheduling node, and one backup node, and 24 data computing nodes. In addition, the corresponding dual-core CPUs with a frequency of 2.5 Ghz and memory up to 8 GB were installed and configured within each node hardware, and the configuration information of the computer software was Hadoop 0.23.0. The training settings are shown in Table 3.

### 4.2. Experimental Results

To verify the effectiveness of the dual-stream network structure and improved residual structure designed in this paper, the subjective evaluation of whether the model of this paper is online teaching form is shown in Table 4.

Table 4 shows that the home-based online teaching format meets most teachers' basic requirements for teaching but is slightly worse in online error correction, interaction, and testing and needs to be improved. Ablation experiments were conducted in the CSL dataset to compare the dual-stream GCN network, GCN+2D-ResNet network, and SCR-GAN network, respectively, with the base GCN network as the baseline, and the experimental results are shown in Figures 5 and 6. The dual-stream GCN network structure has better recognition effect compared with the ordinary GCN network, and the recognition rate is increased by 8%. There is also a considerable increase in accuracy after adding the improved residual structure to the base GCN network, with an increase of 7.3%. Therefore, the improvement of the network in this paper is effective, and the combination of the two approaches greatly improves the recognition accuracy of the network.

To further verify the effectiveness of the proposed SCR-GAN network in gesture recognition, the method is compared with other mainstream methods on two datasets, CSL and DEVISIGN-L, and the results of the comparison experiments are shown in Figures 7–10. From the data in the table, in gesture recognition, the recognition accuracy of the GCN network-based method is significantly higher compared with the CNN network-based method and the RNN network-based method, and the accuracy of the SCR-GAN network on the CSL and DEVISIGN-L datasets reaches 96.2% and 69.3%, respectively, with the highest recognition accuracy and the best recognition effect. The recognition accuracy of both the residual-based DSTA-Net and the dual-stream structure-based 2s-AGCN network is higher, reaching 93.2% and 95.6%, respectively, second only to the network in this paper. The experimental results prove that the combination of residual structure and dual-stream structure can enhance the image sequence extraction ability and make the whole network framework have better generalization ability and recognition effect.

The constructed spatial and temporal maps are used as the input of spatial and temporal flow channels, respectively, to speed up the network training speed, embedding the improved residual structure to increase the network depth and avoiding the problems such as gradient disappearance and converting the sequences output from the two channels in series and feeding them to the input SoftMax classifier to get the final results with good recognition effect. In the future work, we will conduct in-depth research on how to perform accurate recognition under complex conditions such as partial occlusion of hand gestures and continuously optimize the recognition performance of the network.

## 5. Conclusion

The new crown pneumonia epidemic is raging, and overcoming the epidemic is at the same time an opportunity for self-improvement. For the future development trend of online physical education, frontline physical educators should give full play to the advantages of online teaching, learn lessons, and improve deficiencies to further improve the school physical education system and meet the development needs of students in special periods. Online physical education classes are taught with the help of Internet information technology, which breaks the constraints of traditional physical education limited by time and space. Students can choose the right time and place for physical education classes in combination with their own learning arrangements and actual conditions, which improves the autonomy and convenience of physical education class learning. From the perspective of teachers' teaching, online teaching has changed the dilemma that physical education could not be carried out in rainy and snowy weather in the past. In particular, the development of online physical education during the epidemic prevention and control period highlights the necessity of physical education development in special times and triggers thoughts on online physical education in the postepidemic era. The method proposed in this paper effectively addresses closed home physical education, and in the future, we plan to conduct research on closed home physical education models and coping strategies using graph convolutional neural networks.

## Figures and Tables

**Figure 1:** The significance of teaching physical education on the home online.

**Figure 2:** Model structure.

**Figure 3:** Coarse segmentation flow chart.

**Figure 4:** DCNN.

**Figure 5:** Network improvement effectiveness Top-1 verification.

**Figure 6:** Network improvement effectiveness Top-5 verification.

**Figure 7:** Top-1 comparison of different methods on CSL dataset.

**Figure 8:** Top-5 comparison of different methods on CSL dataset.

**Figure 9:** Top-1 comparison of different methods on DEVISIGN-l dataset.

**Figure 10:** DEVISIGN-L Top-5 comparison of different methods on the dataset.

**Table 1:** The development of home online physical education format.

Format	Live %	Videocast %	Communication software %	Other %
Percentage of	37.25	51.12	8.96	2.67

**Table 2:** Convolution block parameter values.

Convolution block parameters	Serial number 1	Serial number 2	Serial number 3	Serial number 4	Serial number 5
Inner core size	7	7	7	7	1
Expansion gap	1	4	16	64	1
Number of channels	16	32	64	128	1

**Table 3:** Training parameters.

Training parameters	Value
Momentum	0.9
Initial learn rate	0.005
Learn rate drop factor	0.5
Learn rate drop period	10
L2 regularization	0.004
Max epochs	50
Minibatch-size	64
Validation frequency	30

**Table 4:** Home online platform format meets basic physical education requirements assessment (%).

Title \ options	Fully satisfied	Satisfied	Basically satisfied	Not satisfied	Did not try
Attendance	46.25	40.78	8.77	0.28	3.92
Explain the knowledge point	65.37	29.27	4.50	0.86	0
Demonstrate movements	89.51	3.21	6.25	1.03	0
Guided practice	55.24	35.30	6.22	1.49	1.75
Online error correction	11.71	24.66	35.45	23.04	5.14
Online interaction	8.22	12.75	31.03	30.25	17.75
Online test and rating	2.50	5.27	18.89	28.60	44.74
Overall rating	9.54	39.48	47.33	3.65	0

## Data Availability

The datasets used during the current study are available from the corresponding author upon reasonable request.
